# Fecal 16S rRNA Gene Sequencing Analysis of Changes in the Gut Microbiota of Rats with Low-Dose Aspirin-Related Intestinal Injury

**DOI:** 10.1155/2021/8848686

**Published:** 2021-04-13

**Authors:** Tianyu Chi, Quchuan Zhao, Peili Wang

**Affiliations:** ^1^Departments of Gastroenterology, Xuanwu Hospital Capital Medical University, Beijing, China; ^2^Cardiovascular Center, Xi Yuan Hospital of China Academy of Chinese Medical Sciences, Beijing, China

## Abstract

**Background:**

The incidence of small intestinal injury caused by low-dose aspirin (LDA) is high, but the pathogenesis and intervention measures of it have not been elucidated. Recent studies have found gut microbiota to be closely associated with onset and development of NSAID-induced intestinal injury. However, studies of the changes in the gut microbiota of rats with LDA-related intestinal injury have been lacking recently. In this study, we investigated fecal 16S rRNA gene sequencing analysis of changes in the gut microbiota of rats with LDA-related intestinal injury.

**Methods:**

Sprague-Dawley (SD) rat models of small intestinal injury were established by intragastric administration of LDA. The small intestinal tissues and the fecal samples were harvested. The fecal samples were then analyzed using high-throughput sequencing of 16S rRNA V3-V4 amplicons. The gut microbiota composition and diversity were analyzed and compared using principal coordinate analysis (PCoA), nonmetric multidimensional scaling (NMDS) analysis, the unweighted pair-group method with arithmetic mean (UPGMA) clustering analysis, multivariate statistical analysis (ANOSIM, MetaStats, and LEfSe), and spatial statistics.

**Results:**

The LDA rat model was successfully established. Decreased Firmicutes and increased Bacteroidetes abundances in rats with LDA-induced small intestinal injury were revealed. MetaStats analysis between the before administration of LDA (CG) and after administration of LDA (APC) groups showed that the intestinal floras exhibiting significant differences (*P* < 0.05, *q* < 0.1) were Firmicutes, Bacteroides, Cyanobacteria, Melainabacteria, Coriobacteriia, Bacteroidia, Bacteroidales, Eubacteriaceae, and Streptococcaceae. In addition, the bacterial taxa showing significant differences between the control (NS) and APC groups were Firmicutes, Bacteroides, Verrucomicrobiaceae and Peptococcaceae.

**Conclusions:**

The alterations in the gut microbiota composition and diversity of rats with LDA-related intestinal injury were found in the present study. The change of gut microbiota in LDA-related intestinal injury will lay the foundation for further research on the function and signaling pathways of the intestinal flora and promote the use of intestinal flora as drug targets to treat LDA-induced small intestinal injury.

## 1. Introduction

Aspirin is the most widely prescribed nonsteroidal anti-inflammatory drug (NSAID) worldwide. Low-dose aspirin (LDA) is widely used in the primary and secondary prevention and treatment of cardiovascular and cerebrovascular diseases. It is estimated that more than two-thirds of regular NSAID users will suffer from small bowel injuries, which are more common than gastroduodenal mucosal lesions. Recent studies suggest that long-term LDA use is associated with lower digestive tract injury and is an important factor in the development of small intestinal ulcers, bleeding, and stenosis. Both short- and long-term LDA use can cause insidious intestinal injury, which occurs in up to 42.1-80% of cases [1, 2]. At present, the available treatment for LDA-related small intestinal injury is unsatisfactory. Although an effective treatment approach is to stop taking aspirin, aspirin withdrawal greatly increases the risks of cardiovascular and cerebrovascular complications and mortality. Some studies have confirmed that misoprostol, metronidazole, and ampicillin can inhibit NSAID-related small intestinal injury [3], but this approach has problems associated with insufficient intestinal protection and poor clinical feasibility. For example, long-term oral antibiotic usage to prevent LDA-related small intestinal injury may cause antibiotic-related bowel disease and antibiotic resistance. Therefore, it is necessary to further investigate the potential mechanism of LDA-related small intestinal injury to promote the prevention and treatment of this type of injury.

Forty years ago, intestinal flora was shown to be involved in NSAID-mediated small intestinal injury. Gnotobiotic rats are resistant to indomethacin-induced intestinal injury, while gnotobiotic rats exposed to Escherichia coli develop severe small intestine damage. Bacterial overgrowth in the small intestine is a major risk factor for NSAID-induced severe intestinal injury [4]. Rifaximin can significantly prevent indomethacin-induced intestinal injury by altering the levels of specific bacterial species [5]. Probiotics and rebamipide can also regulate intestinal flora to prevent NSAID-induced small intestinal injury [6]. Although the results of the abovementioned studies indicate that the intestinal flora plays an important role in NSAID-related small intestinal injury, their effects on LDA-related intestinal injury have not yet been elucidated. Clinical trials have shown that Lactobacillus grigni and Bifidobacterium brevis may help to reduce aspirin-induced injury of the small intestine and relieve gastrointestinal symptoms in humans [7, 8]. However, the specific interplay between LDA-related intestinal injury and intestinal flora as well as the mechanism by which LDA regulates the gut microbiota has remained largely unelucidated. In the present study, Sprague-Dawley (SD) rat models of small intestinal injury were established by intragastric administration of LDA. Subsequently, 16S rRNA V4 region sequencing analysis was conducted on an Illumina HiSeq sequencing platform to investigate the intestinal microecological characteristics of LDA-related small intestinal injury and to elucidate the mechanism associated with intestinal flora imbalance in LDA-related small intestinal injury.

## 2. Materials and Methods

### 2.1. Drugs, Reagents, and Instruments

Bayaspirin enteric-coated tablets (0.1 g/tablet, Bayer Medical Care, Germany) were used in the present study. Based on the long-term oral aspirin dose (100 mg/d) used in humans, the administered rat aspirin dosage was 10.41 mg/kg/d (dissolved in 50 ml 0.9% sodium chloride solution), and the prepared LDA solution was stored in a refrigerator at 4°C. DSS (MP Biomedicals, USA, batch number: 18008540530), an E.Z.N.A. Stool DNA Kit (Omega Bio-Tek, USA), a TruSeq® DNA PCR-Free Sample Preparation Kit, 16S V3-V4 region primers (338F and 806R), an Illumina MiSeq PE250 sequencing platform (Illumina, USA), 2% agarose gel, a CFX96 PCR instrument (Bio-Rad, USA), Leica EG1150H embedding machine (Leica, Germany), an Excelsior ES dehydrator (Somerfly, USA), and a Leica RM2245 microtome (Leica, Germany), CX31 microscope (Olympus, Japan) were all used in the present study.

### 2.2. Preparation and Grouping of Animal Models

Six male SD rats aged 6-7 weeks and weighing 200-220 g were used in the present study and provided by Beijing Huafukang Biotechnology Co., Ltd. (animal certificate number: SCXK (Beijing) 2019-0008 (license number)). The temperature of the feeding environment was maintained at 24 ± 1°C, and the humidity was 45 ± 15%. Six rats were divided into the LDA group (3 rats) and the control group (3 rats) using the random number table method. The rats were regularly provided food and water, and their bedding was frequently changed to maintain the cleanliness of the animals. Fecal specimens from rats in the LDA group before treatment were retained for subsequent analysis. Two groups of rats were treated by gavage at the same time each day as follows: for the control group, 1 ml of 0.9% sodium chloride solution was infused into the stomach of each rat once a day using an intragastric needle, and normal water was provided for 14 days; and for the LDA group, based on the weights of the rats, the prepared LDA solution was infused into the stomachs of rats once a day by intragastric needle, and normal water was provided for 14 days. No dead animals appeared during the modeling period. All animal experiments performed in the present study complied with relevant national animal ethics and welfare regulations and requirements.

### 2.3. Animal Sample Materials

The procedures for fecal sample collection are as follows: after the last administration of drugs to the rats on the 14th day, the rats were fasted and treated with water for 24 h. After perianal disinfection, the rats were urged to defecate by abdominal massage. Then, 2-4 capsules or 1-2 ml of feces was collected with sterile forceps and stored in sterile cryopreservation tubes at -80°C for subsequent fecal DNA extraction and bacterial flora detection. The procedures for small intestinal tissue collection are as follows: after fecal sample collection, all rats in each group were sacrificed, and small intestinal tissues were dissected and stored in 4% neutral formaldehyde for subsequent histopathological evaluation.

## 3. Methods

### 3.1. Histopathological Evaluation

The jejunum and ileum of each rat were dissected. Then, the contents of the intestinal cavity were washed with buffer 3 times, after which the ulcer was measured with a Vernier caliper. The degree of small intestinal injury was scored according to the Reuter scoring method (Tables 1 and 2), and the results were scored as the sum of the ulcer and adhesion indices. Small intestinal tissue blocks were obtained from the most obvious site of injury, portions of which were then fixed with neutral formic acid buffer. Conventional dehydration and paraffin embedding were performed to generate 4 *μ*m thick sections. Subsequently, pathological sections were obtained by HE staining and fixation, and the pathological tissues were then observed under a light microscope. The degree of small intestinal injury was evaluated according to Chiu's criteria (0-4 scale), where 0 points denotes normal intestinal mucosal villi; 1 point denotes the occurrence of cystic spaces under the epithelium at the top of the villi with capillary congestion; 2 points denotes an enlarged subepithelial space, a moderate lamina propria edema, and a dilated central chyle duct; 3 points denotes an obvious edema of the lamina propria, degeneration and necrosis of the epithelial layer of the intestinal mucosa, and a little villus tip shedding; and 4 points denotes degeneration and necrosis of the epithelial cell layer, some villi shedding, naked lamina propria, and telangiectasia.

### 3.2. Fecal DNA Extraction and PCR Amplification and Purification

Each fecal sample (200 mg) was aseptically weighed and transferred to a 2 ml Ep tube. Then, fecal DNA was extracted using a PowerSoil DNA Isolation Kit (MoBio Laboratories, Carlsbad, CA) and assessed for DNA quality and concentration using a NanoDrop fluorospectrometer. Subsequently, an appropriate amount of each sample was transferred into separate centrifuge tubes and diluted to 1 ng/*μ*l with sterile water. The diluted genomic DNA samples were used as template for PCR amplification using specific barcoded primers. After detection of the products by 1% agarose gel electrophoresis, the PCR products were purified using an automated magnetic bead method.

### 3.3. Library Construction and High-Throughput Sequencing

Libraries were constructed with a Library-Building Kit and quantified using a Qubit instrument and by qPCR. Then, 16S rRNA gene V3-V4 sequencing was performed on an Illumina MiSeq platform after the MiSeq library passed quality inspection.

### 3.4. Sequence Analysis

After the original sequencing data was downloaded, quality control steps were performed, and the optimized sequences were obtained by sequence splicing, filtering, and dechimerization. Then, the operational taxonomic units (OTUs) were clustered and annotated at a 97% similarity threshold. Alpha and beta diversity analyses were performed based on the clustering results. In addition, based on the annotation results, the classification information at each level could be obtained, and the correlation analysis of sample composition and community structure differences between samples could also be conducted.

## 4. Statistical Methods

QIIME was used to compare sample complexity and diversity in the present study. Basic analysis of OTUs was performed, including the generation of a Venn diagram of OTU distribution and OTU cluster analysis. Species annotation was based on the OTUs and the taxonomic heat map analysis. Rank-abundance and Shannon indices were used to evaluate the total number and diversity of bacterial species. Principal coordinate analysis (PCoA), which is similar to PCA analysis, was performed to study the similarities or differences in sample community composition. Nonmetric multidimensional scaling (NMDS) analysis was performed using the weighted UniFrac distance algorithm, and two coordinate axes that could reflect the differences between samples to the greatest extent were selected for graphical display by dimension reduction of the multidimensional data. In addition, a sample clustering tree was constructed using the unweighted pair-group method with arithmetic mean (UPGMA) clustering analysis to study the similarity of the floral composition among different samples, and the clustering results were integrated with the relative abundance of species of each sample at the different levels. To further assess the differences in community structure among the groups, three multivariate statistical analysis methods (ANOSIM, MetaStats, and LEfSe) were used to test the significance of differences in species composition and community structure between the groups and to identify the species with significant differences at all levels. Network analysis results clearly showed the interaction between intestinal floras.

## 5. Results

### 5.1. Gross Pathology Changes in Small Intestinal Mucosa

No small intestinal mucosal injury was detected in the control group. The mucosa of the small intestine remained intact, and no swelling, erosion, bleeding, and bowel adhesion were observed. After intragastric administration of LDA, scattered punctate erosion was observed in the small intestinal mucosa of rats, and a small amount of sheet erosion was detected throughout the entire small intestine. Part of the small intestine adhered to the adjacent intestine, yet it could be stripped with light force. The average gross injury scores of small intestinal mucosa in the control and LDA groups were 0.000 and 2.667, respectively, indicating that the small intestinal mucosa was damaged in the LDA group.

### 5.2. Histological Staining Changes of Small Intestinal Mucosa

In the control group, the morphology of the small intestinal mucosa was normal, the villi were arranged regularly, the epithelial layer was intact, and the top was not damaged. In the LDA group, we observed that villi and glandular epithelium atrophied in the mucosa of the small intestine, cystic spaces appeared in the tops of villi with monocytes infiltrating in the surface layer, and the epithelial layer was incomplete. The LDA group exhibited remarkable inflammatory reactions compared with the control group, which indicated that intestinal mucosal injury in the LDA rat models was successfully established (see Figure 1). The average histological injury scores of small intestinal mucosa in the control and LDA groups were 0.000 and 2.333, respectively.

The control group (Figure 1(a)) exhibited scattered infiltration of lymphocytes, and eosinophils were detected in the stroma of intestinal mucosa. The LDA group (Figure 1(b)) exhibited local surfaces of the small intestinal mucosa that were eroded, and a large amount of lymphocyte infiltration was observed in the muscular layer of the mucosa accompanied by lymphoid tissue hyperplasia and lymphoid follicle formation.

## 6. Changes in the Gut Microbiota of Rats with LDA-Induced Small Intestinal Injury

To characterize the microbiota of the study rats, we collected nine fecal samples, including from the control group (NS group, *N* = 3) and the LDA group before (CG group, *N* = 3) and after administration of LDA (APC group, *N* = 3). DNA was purified from each sample and then used as template for 16S rRNA V3-V4 gene tag amplification and sequencing.

### 6.1. OTU Analysis

#### 6.1.1. OTU Distribution for the Three Groups

Three samples in each group were sequenced to obtain OTU data, which is presented in a Venn diagram (Figure 2). Bioinformatics analysis was performed to group sequences into OTUs at a >97% similarity threshold, resulting in 783 OTUs being detected in the three groups. After leveling, 740 OTUs were identified, 352 of which were detected in all three groups.

Seven hundred eighty-three OTUs were detected in the three groups. After leveling, 740 OTUs remained, 352 of which were detected in all three groups.

#### 6.1.2. Relative Abundances of Intestinal Flora

No significant differences between the intestinal flora at the phylum, class, order, family, and genus levels were observed between the NS and CG groups. However, differences in microflora composition were detected between the CG and APC groups. The dominant phyla, including Firmicutes and Bacteroidetes, showed significant differences after LDA treatment, including decreased Firmicutes and increased Bacteroidetes abundances. Differences in OTU abundance between groups were analyzed at the phylum, class, order, and family levels using histograms (Figure 3).

At the phylum level, the proportion of Firmicutes in the APC group was significantly lower than that observed in the CG group, while the proportion of Bacteroidetes in the APC group was significantly higher than that detected in the CG group (Figure 3(a)). At the class level, the proportion of Clostridia in the APC group was significantly lower than that observed in the CG group, while the proportion of Bacteroidia in the APC group was significantly higher than that detected in the CG group (Figure 3(b)). At the order level, the proportion of Clostridia in the APC group was lower than that observed in the CG group, while the proportion of Bacteroidales in the APC group was significantly higher than that detected in the CG group (Figure 3(c)). At the family level, the proportion of Lachnospiraceae in the APC group was lower than that observed in the CG group, while the abundance of Bacteroidales_S24-7 in the APC group was significantly higher than that detected in the CG group (Figure 3(d)).

#### 6.1.3. Heat Map Analysis

A clustering analysis of species abundance similarity among the samples was performed, and the results are presented in a heat map (Figure 4). The abundances of Bacteroidetes, Clostridia, Lachnospiraceae, and Bacteroidales_s24-7 were apparently higher in the APC group than in the CG group.

Higher abundances of Bacteroidetes (phylum level; Figure 4(a)), Bacteroidia, and Clostridia (class level; Figure 4(b)); Clostridiales and Bacteroidales (order level; Figure 4(c)); and Lachnospiraceae and Bacteroidales_s24-7 (family level; Figure 4(c)) were observed in the APC group than in the CG group.

#### 6.1.4. Sample Clustering Histogram

Based on an unweighted UniFrac distance matrix, the UPGMA method was used to cluster the samples, and the results were compared to the relative abundances of each sample at the phylum, class, order, family, and genus levels. The results demonstrated that the three samples in the APC group clustered well (Figure 5).

APC1 and APC3 clustered well with respect to richness at the phylum level (Figure 5(a)); APC2 and APC3 clustered well at the class level (Figure 5(b)); APC2 and APC3 clustered well at the order level (Figure 5(c)); and APC1 and APC2 clustered well at the genus level (Figure 5(d)).

### 6.2. Alpha Diversity Analysis

Based on the alpha diversity indices of the three groups, including Chao1, observed_species, and Shannon, no significant differences were detected in pairwise comparisons (*P* > 0.05).

### 6.3. Beta Diversity Analysis

#### 6.3.1. PCoA and PCA

Based on the PCoA and NMDS, the floral composition of the APC group was significantly different from that of the CG and NS groups, while the bacterial composition of the CG and NS groups was similar. According to the PLS-DA results, the relationship between different microbial contents and different groups indicated that different microbial contents could be used to predict different sample types (Figure 6).

#### 6.3.2. ANOSIM

ANOSIM was used to test whether differences between groups (two or more groups) were significantly greater than those within groups (Table 3). ANOSIM showed significant and remarkable differences among the three groups (*P* = 0.016, *P* < 0.05). Although not significantly different, the *R*-values for the CG-APC and NS-APC comparisons were all greater than zero (0.5185 and 0.4444, respectively), indicating potential differences between the CG and APC groups and the NS and APC groups.

#### 6.3.3. MetaStats Test

The results of the MetaStats analysis between the CG and APC groups showed that the intestinal floras exhibiting significant differences (*P* < 0.05, *q* < 0.1) were Firmicutes, Bacteroides, Cyanobacteria, Melainabacteria, Coriobacteriia, Bacteroidia, Bacteroidales, Eubacteriaceae, and Streptococcaceae (Table 4). In addition, the bacterial taxa showing significant differences between the NS and APC groups were Firmicutes, Bacteroides, Verrucomicrobiaceae, and Peptococcaceae (Table 5). No significant differences in flora were observed between the NS and CG groups at the phylum, class, order, family, and genus levels.

#### 6.3.4. LEfSe

Among the three groups, the abundances of Rhodospirillales, Rhodospirillaceae, and Alphaproteobacteria in group APC were significantly different from the other two groups. The abundances of Firmicutes, Anaerofustis, and Eucharacteriacea in the CG group were significantly different from those observed in the other two groups. The abundance of Papillibacter in group NS was significantly different from that observed in the other two groups (Figure 7).

### 6.4. Network Analysis

Through Spearman network analysis, the top 20 OTUs with the greatest absolute abundances among all samples were selected for correlation analysis at the phylum level. The calculated results were plotted after filtering out differences with a *P* value greater than 0.05 or a correlation coefficient ∣*R* | <0.4 (Figure 8).

## 7. Discussion

Gut microbes play an important role in host physiology, pathology, and intestinal immune balance. In the present study, Bacteroidetes and Firmicutes dominated the rat intestinal flora, followed by Proteobacteria and Actinomycetes. In previous experiments, high-throughput sequencing has been used to analyze the intestinal flora of rats, with the results showing that the composition of the intestinal flora of normal rats is similar to that of human intestinal flora. Aspirin can lead to an imbalance of the intestinal flora, destroy the intestinal mucosal barrier, and produce pathological changes similar to aspirin-induced human intestinal injury in animal models. The changes in the intestinal flora resulting from LDA-induced small intestinal injury were investigated in the present study. During model replication, the rats showed histopathological changes similar to those observed during aspirin-induced injury of the human intestinal tract. In our present study, bacterial flora analysis suggested that the abundance of Firmicutes decreased and that of Bacteroides increased in the rat models of LDA-induced small intestinal injury.

Intestinal bacteria are key factors in NSAID-induced intestinal inflammation that play a dual role in the pathogenesis of NSAID-induced intestinal injury by participating in the hepatointestinal circulation of NSAIDs and activating the innate immune system. Recent microbiome analyses have shown that NSAIDs can cause the dysbiosis of various intestinal floras in the small intestine, including increases in the abundances of some gram-negative bacteria, such as Clostridium [9] and Enterococcus [10]. Furthermore, gram-negative bacteria (e.g., Escherichia coli and members of the phylum Proteobacteria) play a crucial role in the development of small intestinal ulcers. Previous studies have shown that NSAIDs can cause an increase in the number of gram-negative bacteria in the small intestine during the development of injuries [11, 12]. Indomethacin treatment can promote an increased proportion of gram-negative bacteria in the gut, including c-Proteobacteria and Bacteroidetes [13]. However, the results of the present study showed that LDA-induced changes in enterobacteria were different from those mediated by other types of NSAIDs. At the phylum level, the proportion of Bacteroidetes and Verrucomicrobia decreased and that of Cyanobacteria increased during indomethacin-induced small intestinal injury, whereas in the LDA group, the same changes in Verrucomicrobia and Cyanobacteria were observed, while the proportion of Bacteroidetes increased in the LDA group. The proportion of Firmicutes increased during indomethacin-induced small intestinal injury but was decreased in the LDA group. In addition, the proportion of Proteobacteria increased during indomethacin-induced small intestinal injury, while no significant changes were observed in the LDA group. At the genus level, the abundance of Streptococcaceae increased during indomethacin treatment but was decreased in the LDA group. Changes in the small intestinal microbiota, increased mRNA levels of inflammatory cytokines, and greater numbers of small intestinal ulcers were also observed to occur almost simultaneously during indomethacin-induced small intestinal injury, and the changes in intestinal microbiota were somewhat prolonged even when the ulcer was cured [14].

Previous studies on intestinal flora in NSAID-related enteropathy support the conclusions of the present study to some extent. Diclofenac has been shown to reduce ileal occludin expression and increase the abundance of Proteobacteria and Bacteroidetes in the intestinal flora, and the results of the present study also showed that LDA increased the abundance of Bacteroidetes in the intestine. Thus, rifaximin can prevent diclofenac-induced enteropathy through its antimicrobial and anti-inflammatory effects [15]. A study in humans revealed that the total number of microorganisms in elderly individuals taking NSAIDs was higher than that observed in individuals not taking NSAIDs [16]. In a 16S rRNA gene sequence analysis, the abundance of Firmicutes decreased while that of Bacteroidetes increased in elderly individuals taking NSAIDs, which is in complete agreement with the conclusions of the present study. At the genus level, the proportion of butyrate-producing Clostridium cluster XIVa, members of which include Roseburia and Ruminococcus, was observed to be reduced in elderly individuals taking NSAIDs. In addition, the abundance of Lactobacillus was observed to be significantly lower in elderly subjects taking NSAIDs than in those not taking drugs. In general, a decrease in the abundance of Firmicutes and changes in the function of the intestinal epithelium can have a significant impact on human intestinal health. One study on the mucosal microbiota in patients with inflammatory bowel disease showed a decrease in Firmicutes (especially Roseburia and Faecalibacterium prausnitzii) and an increase in Proteobacteria and Actinobacteria compared to healthy controls [17].

However, the conclusions of the present study are also contradictory to those of previous studies with respect to the effects of some types of NSAIDs on the intestinal flora. A previous study showed that the levels of inflammation and tissue peroxidation markers were remarkably increased in the jejunum and ileum of indomethacin-treated rats, which could cause alterations in the intestinal microbiota, including increased Firmicutes and decreased Bacteroidetes abundances [18]. However, in rats treated with rifaximin-EIR, the intestinal microbiota was not significantly different from that observed in those of the control group, and rifaximin-EIR was also able to counteract the increased abundance of Proteobacteria and Firmicutes caused by indomethacin. Thus, rifaximin-EIR treatment significantly inhibits the intestinal injury induced by indomethacin, and this intestinal protective effect is associated with reduced tissue inflammation, oxidative stress and gastrointestinal bleeding, and the reversal of bacterial population changes caused by NSAIDs [5, 19]. In a human trial of dual antiplatelet therapy (DAPT), the intestinal flora of the aspirin and clopidogrel group was significantly different from that of the control group at the class, order, family, and genus levels, although DAPT did not cause changes in the biodiversity of the intestinal flora [20]. The DAPT group showed a higher abundance of Bacilli and a lower abundance of Erysipelotrichia at the class level; a higher abundance of Lactobacillales and lower abundance of Erysipelotrichales at the order level; a higher abundance of Streptococcaceae and Lactobacillaceae and a lower abundance of Acidaminococcaceae and Erysipelotrichaceae at the family level; and a higher abundance of Streptococcus and Klebsiella and a lower abundance of Blautia, Phascolarctobacterium, and Megamonas at the genus level.

In situ, within the deep layers of the ileum in Crohn's disease patients with ileocecal resection, researchers observed that the abundances of Bacteroidetes and Clostridia in Crohn's disease patients were significantly decreased compared to those observed in the normal group [21]. The results of our present study also indicated that the abundance of Clostridia was remarkably decreased in rats with LDA-induced small intestinal injury, whereas that of Bacteroides was increased. Lachnospiraceae are abundant obligate anaerobic bacteria in the human intestine that affects host health by producing short-chain fatty acids, participating in bile acid metabolism, and promoting colonization resistance against intestinal pathogens. Members of the family Lachnospiraceae have been well studied in inflammatory bowel disease. A previous study reported that disorders of the protective gut commensal strain network, including the families Lachnospiraceae and Ruminococcaceae, which produce short-chain fatty acids, are associated with the frequent recurrence of inflammatory bowel disease and poor response to treatment with anti-TNF-*α* antibodies [22]. The results of the present study showed that the abundance of Lachnospiraceae decreased in the LDA-induced small intestinal injury rats and that Ruminococcaceae interacted with the most bacteria in the intestine, suggesting that they may have an effect on LDA-induced small intestinal injury. In the mouse model of dextran sodium sulfate-induced colitis, the abundance of Bacteroidales_S24-7 family and short-chain fatty acid-producing bacteria was shown to be lower [23]. Nevertheless, the results of the present study showed that the abundance of the Bacteroidales_S24-7 family was increased in rats with LDA-induced small intestinal injury. The relative abundance of Alphaproteobacteria (order RF32) was shown to be positively correlated with the histopathology of damaged colon and colonic inflammation in mice with Crohn's disease [24], and a high abundance of this taxon was also observed during LDA-induced small intestinal injury. A correlation analysis performed in another study showed that proinflammatory cytokines and other injury-related factors were negatively correlated with Verrucomicrobia and Ruminococcaceae in inflammatory bowel disease model mice [25]. The abundance of Verrucomicrobia was significantly decreased in rats with LDA-induced small intestinal injury compared to that observed in the control group in the present study. Interestingly, Ruminococcaceae has been shown to be one of the most differentially abundant bacterial taxa between individuals with inflammatory bowel disease and healthy controls [17, 26]. In the present study, Ruminococcaceae was also observed to interact with the most bacteria in the intestine and may be involved in the small intestinal inflammatory response induced by LDA.

To achieve more reliable and comprehensive results, we believe that the following additional experiments should be performed. First, this study is a preliminary experiment with a small sample size, and the results of the study have certain limitations. In order to verify the accuracy of the results, we need to further expand the sample size to verify the experimental results in the future experiments. Secondly, a metagenomics analysis should be performed to further determine the function and important signaling pathways of the intestinal flora identified as being important in LDA-induced small intestinal injury. Then, fecal bacterial transplantation experiments should be performed in gnotobiotic rats using feces from LDA rat models [27]. Finally, it is necessary to expand the sample size and to detect the levels of relevant inflammatory factors and short-chain fatty acids to further investigate the pathogenesis of LDA-induced small intestinal injury.

The results of previous studies have suggested that probiotics play a significant role in intestinal inflammatory diseases through multiple aspects [28]. Probiotics compete with pathogenic microorganisms for nutrients and produce bacteriostatins to effectively prevent pathogenic microorganisms from invading and reproducing in the intestine [29]. Furthermore, probiotics can synthesize short-chain fatty acids (SCFAs) that can be used for energy by the colonic epithelium, and SCFAs can regulate cellular and humoral immunity, especially gut mucosa-associated lymphoid tissue (GALT) [30, 31]. Probiotics can also inhibit the growth of pathogens by reducing the intestinal pH and can also directly supplement beneficial flora or stimulate their growth. In addition, probiotics prevent bacteria from adhering to intestinal epithelial cells, thereby preventing pathogenic bacteria from crossing the intestinal mucosal epithelial barrier and blocking bacterial migration [32]. Probiotics are also useful as a preventive measure to alleviate intestinal inflammation, and because they increase the surface area of the villi in the small intestine, probiotics promote nutrient absorption. Probiotics are typically used in the treatment of intestinal diseases due to their natural, safe, and effective properties compared to traditional drugs [33, 34]. However, the role of probiotics in the prevention and treatment of LDA-induced small intestinal injury is controversial. Therefore, identifying probiotic formulations suitable for LDA patients is an important goal of future research. The results of this study and subsequent studies will provide insights for future efforts to target the microbiota as a therapeutic strategy and provide a foundation for clinical application of probiotics in the prevention and treatment of LDA-induced small intestinal injury.

## 8. Conclusions

In the present study, we observed decreased Firmicutes and increased Bacteroidetes abundances in rats with LDA-induced small intestinal injury through 16S rRNA gene sequencing analysis. At the phylum level, the proportion of Firmicutes in the LDA group was significantly lower than that observed in the preadministration group, while the proportion of Bacteroidetes in the LDA group was significantly higher than that detected in the preadministration group. At the class level, the proportion of Clostridia in the LDA group was significantly lower than that observed in the preadministration group, while the proportion of Bacteroidia in the LDA group was significantly higher than that detected in the preadministration group. At the order level, the proportion of Clostridia in the LDA group was lower than that observed in the preadministration group, while the proportion of Bacteroidales in the LDA group was significantly higher than that detected in the preadministration group. At the family level, the proportion of Lachnospiraceae in the LDA group was lower than that observed in the preadministration group, while the proportion of Bacteroidales_S24-7 in LDA group was significantly higher than that observed in the preadministration group. The results of the present study will lay the foundation for further research on the function and signaling pathways of the intestinal flora and promote the use of intestinal flora as drug targets to treat LDA-induced small intestinal injury.

## Figures and Tables

**Figure 1:** HE staining of the small intestinal mucosa in two groups (10x magnification).

**Figure 2:** Venn diagram of the distribution of OTUs in the three groups.

**Figure 3:** Analysis of OTU abundance at the phylum, class, order, and family levels.

**Figure 4:** Heat map of bacterial abundance in the three groups.

**Figure 5:** Clustering of the nine samples.

**Figure 6:** PCoA and PCA. (a) PCoA plot based on Bray-Curtis dissimilarity. The APC, CG, and NS groups could be effectively separated, indicating that the composition of the intestinal flora in the APC group was significantly different from that of the CG and NS groups. However, the CG and NS groups were not effectively separated, indicating that the gut bacterial compositions of the two groups was similar. (b) NMDS at OTU level analyses. No intersection between the APC group and the CG and NS groups was observed, demonstrating that the APC group was different from the CG and NS groups. In contrast, an intersection between the CG and NS groups was observed, demonstrating that there was no significant difference between these groups. (c) PLS-DA analysis based on OTUs. The APC, CG, and NS samples were effectively separated, and the relationships between different microbial contents and groups indicated that different microbial contents could be used to predict different groups.

**Figure 7:** LDA distribution of LEfSe results based on the classification information. The threshold value of the LDA score was set to 3, and an LDA score >3 was considered significant. The abundances of Rhodospirillales, Rhodospirillaceae, and Alphaproteobacteria in group APC were significantly different from those observed in the other two groups. The abundances of Firmicutes, Anaerofustis, and Eucharacteriacea in group CG were significantly different from those observed in the other two groups. The abundance of Papillibacter in group NS was significantly different from that observed in the other two groups.

**Figure 8:** Cooccurrence network of intestinal flora. Ruminiclostridium and Roseburia, members of the phylum Firmicutes, exhibited the most interactions with other bacteria.

**Table 1:** Reuter scoring criteria for the small intestinal ulcer index in rats.

Ulcer score	0	1	2	3	4	5
Ulcer degree	No ulceration	Local congestion, no ulcer	Ulcers without congestion or intestinal wall thickening	Ulcers and inflammation in 1 site	Ulcers or inflammatory reactions in 2 or more sites	Perforation

**Table 2:** Reuter scoring criteria for the small intestinal adhesion index in rats.

Adhesion score	0	1	2
Adhesion degree	No adhesion	Light adhesion (slightly forceful separation of the small intestine from other tissues)	Heavy adhesion

**Table 3:** ANOSIM results.

Group	*R* statistic	*P* value	Number of permutations
CG-NS	0.1111	0.297	999
CG-APC	0.5185	0.103	999
NS-APC	0.4444	0.095	999
All	0.3663	0.016	999

**Table 4:** Intestinal flora showing significant differences (*P* < 0.05, *q* < 0.1) between the CG and APC groups in the MetaStats test.

	Intestinal flora	CG group (mean ± SD)	APC group (mean ± SD)	*P* value	*Q* value
Phylum	Firmicutes	0.763803 ± 0.071358	0.485976 ± 0.055749	0.010	0.024
	Bacteroidetes	0.207045 ± 0.067676	0.467576 ± 0.038210	<0.001	<0.001
	Cyanobacteria	0.000082 ± 0.000000	0.004289 ± 0.002449	0.020	0.032
Class	Melainabacteria	0.000082 ± 0.000000	0.004289 ± 0.002449	0.011	0.069
	Coriobacteriia	0.012737 ± 0.004690	0.003701 ± 0.004690	0.022	0.090
	Bacteroidia	0.207045 ± 0.067676	0.467353 ± 0.038105	<0.001	<0.001
Order	Bacteroidales	0.207045 ± 0.067676	0.467353 ± 0.038105	<0.001	<0.001
Family	Eubacteriaceae	0.000399 ± 0.000000	0.000012 ± 0.000000	<0.001	<0.001
	Streptococcaceae	0.001175 ± 0.000000	0.000059 ± 0.000000	0.003	0.088

**Table 5:** Intestinal flora showing significant differences (*P* < 0.05, *q* < 0.1) between the NS and APC groups in the MetaStats test.

	Intestinal flora	NS group (mean ± SD)	APC group (mean ± SD)	*P* value	*Q* value
Phylum	Firmicutes	0.661873 ± 0.073471	0.485976 ± 0.055749	0.019	0.023
	Bacteroidetes	0.258063 ± 0.134666	0.467576 ± 0.038210	0.048	0.038
	Verrucomicrobia	0.011891 ± 0.001732	0.000564 ± 0.000000	0.009	0.021
Class	Verrucomicrobiae	0.011891 ± 0.001732	0.000564 ± 0.000000	<0.001	<0.001
Order	Verrucomicrobiales	0.011891 ± 0.001732	0.000564 ± 0.000000	<0.001	<0.001
Family	Peptococcaceae	0.006380 ± 0.001000	0.000952 ± 0.001000	0.003	0.060
	Verrucomicrobiaceae	0.011891 ± 0.001732	0.000564 ± 0.000000	<0.001	<0.001

## Data Availability

The data used to support the findings of this study are included within the article.
